The article "Hemodynamic Impact of Stenting on Carotid Bifurcation: A Potential Role of the Stented Segment and External Carotid Artery" was published in 2021. Journal: Comput Math Methods Med.

# Hemodynamic Impact of Stenting on Carotid Bifurcation: A Potential Role of the Stented Segment and External Carotid Artery

**DOI:** 10.1155/2021/7604532

**Published:** 2021-11-26

**Authors:** Zhenmin Fan, Xiao Liu, Yingying Zhang, Nan Zhang, Xia Ye, Xiaoyan Deng

**Affiliations:** ^1^School of Mechanical Engineering, Jiangsu University of Technology, Changzhou Jiangsu 213001, China; ^2^Key Laboratory for Biomechanics and Mechanobiology of Ministry of Education, School of Biological Science and Medical Engineering, Beihang University, Beijing 100191, China; ^3^Beijing Key Laboratory of Rehabilitation Technical Aids for Old-Age Disability, National Research Center for Rehabilitation Technical Aids, Beijing 100176, China; ^4^Radiologic Department, Beijing Anzhen Hospital, Capital Medical University, Beijing 100029, China

## Abstract

Carotid stenting near the bifurcation carina is associated with adverse events, especially in-stent restenosis, thrombosis, and side branch occlusion in clinical data. This study is aimed at determining the potential biomechanical mechanisms for these adverse events after carotid stenting. The patient-specific carotid models were constructed with different stenting scenarios to study the flow distribution and hemodynamic parameters, such as wall shear stress (WSS), flow velocity, relative residence time (RRT), and oscillating shear index (OSI) in the carotid bifurcation. The results suggested that the existing stents surely reduced blood flow to the external carotid artery (ECA) but enhanced local flow disturbance both in ECA and stented internal carotid artery (ICA), and the inner posterior wall of the stented ICA and the outer posterior wall of ECA might endure a relatively low level of WSS and remarkably elevated OSI and RRT. In addition, the implanted stent leads to more ECA adverse flow than ICA after stenting. While disturbed flow near the strut increased as stent length increased, blood flow and areas of local flow disturbance in ECA slightly decreased as stent length increased. In conclusion, the results revealed that ECA might be in relatively high levels of abnormal local hemodynamics after stenting, followed by stented ICA, leading to potential adverse events after intervention.

## 1. Introduction

The carotid bifurcation consists of the external carotid artery (ECA), internal carotid artery (ICA), and common carotid artery (CCA). Early clinical studies demonstrated that atherosclerotic lesions in the carotid bifurcations usually developed at the distal CCA and the proximal ICA [1–3]. As a breakthrough treatment for occlusive vascular disease, the intervention becomes an effective and widely used option, especially for carotid bifurcation lesions. However, this treatment may account for clinical events during follow-up. The disadvantages of this treatment are clinically evidenced by a relatively high risk of in-stent recurrent stenosis and the fatal complication of in-stent thrombosis [4–6]. In-stent restenosis (ISR) after stenting in the carotid has been stated to range from 1% to 50%, with worse patient outcomes in the long run due to postoperative complications [1, 4–6]. Moreover, intervention for carotid bifurcation is an independent predictor for occlusion of branches without stenting. The implanted stent usually covers the segment of ICA or CCA because of atherosclerotic lesions. Interestingly, ipsilateral ECA after stenting at the carotid bifurcation presents a high risk of occlusive disease [1–3]. The trial included 312 patients in Netherlands and found that more than 50% of stenosis in ipsilateral ECA emerged after carotid stenting [7]. These clinical data suggested that the carotid bifurcation intervention technique caused clinical events at the stented segment and had adverse effects on the branches without stenting. Both of these impacts of stenting on the host artery may lead this treatment to compromised clinical benefits.

The article "Hemodynamic Impact of Stenting on Carotid Bifurcation: A Potential Role of the Stented Segment and External Carotid Artery" was published in 2021. Journal: Comput Math Methods Med.

Despite the complicated and multifactorial reasons for these adverse events, the changed hemodynamics caused by stenting has an essential role in the procession of adverse in-stent events and the ipsilateral branch occlusion [8–10]. The implanted stent certainly disturbs the local blood flow in the host artery and causes flow separation and stagnation flow around the stent struts, manifested by high relative residence time (RRT) and oscillating shear stress index (OSI), but low wall shear stress (WSS) [11–13], which are evidenced to contribute the vascular injury and ISR and stent thrombosis [8–10]. Since little information is available both on the stented vessel and other branches of bifurcations after stenting, we herein aimed to investigate a potential role of intervention in ECA and stented ICA, based on images of in vivo human patient-specific carotid bifurcation. As non-Newtonian and pulsatile behaviors of blood flow, this work analyzed the local hemodynamic conditions of carotid bifurcation after ICA stenting in terms of velocity field, flow distribution, WSS, OSI, and RRT. The impact of stenting scenarios (long, medium, and short stenting) on the hemodynamic performance of the treated carotid bifurcation was also addressed.

## 2. Methods

### 2.1. Image-Based Computational Model after Carotid Stenting

The patient-specific carotid bifurcation with stenosis (Figure 1(a)) was constructed based on angiographic images at some point of the cardiac cycle. In the present study, a total of 323 contiguous carotid artery slices were captured by an imager (Siemens Medical Solutions, Forchheim, Germany) with a voxel size of 2.54 × 2.54 × 5 mm^3^. The carotid bifurcation images in this study included ICA, ECA, and CCA. As shown in Figure 1(a), ICA and CCA were 68 mm and 71 mm at least in length for the more extensive and accurate numerical results [14, 15]. An eccentric type of stenosis was observed, and the narrowest luminal stenosis rate of ICA was 78.5%.

The article "Hemodynamic Impact of Stenting on Carotid Bifurcation: A Potential Role of the Stented Segment and External Carotid Artery" was published in 2021. Journal: Comput Math Methods Med.

After the scanning, the lumen boundaries of the carotid bifurcation were manually segmented by Mimics (Materialise N.V.) to develop the carotid model, while the centerline of the carotid was simultaneously exacted. The constructed model was verified by automated detection using watershed transform from markers [17, 18]. The initial rough geometry (Figure 1(a)) was smoothed slightly in Geomagic (Geomagic, 2013, North Carolina, USA). This study was carried out following Beijing Anzhen Hospital regulations, and all volunteers approved this study and written informed consent.

The commercial carotid stent, whose structures resemble the reported ViVEXX, was constructed by Pro/E (Parametric Technology Corporation). Strut thickness of the stent is 81 *μ*m. Extensive details about the geometrical parameters of the stent can be found in early works [19].

The stent was finally assembled in the diameter reduction region along the lumen centerline by Pro/E, while the stenosis was removed from the carotid model. Each stent totally covered the region of lesion, and due to variations in target artery size, the diameter of stent to artery ratio ranged from 1 : 1 to 1.2 : 1 [20]. Since clinical evidences showed that long stent was significantly related to restenosis [21–23], the impact of stent length on hemodynamics after stenting was carried out in the present study. Carotid models 2-4 (Figures 1(b)–1(d)) were investigated numerically with short (13.2 mm), medium (17.7 mm), and long (22 mm) stenting, respectively.

### 2.2. Numerical Approaches

*Assumptions*: we assumed that blood was a kind of non-Newtonian and homogeneous fluid [24, 25].

*Governing equations*: numerical simulations for blood flow and drug were carried out based on Navier-Stokes equations and mass transport equation [26, 27].

(1) $$\begin{array}{c} \rho \left(\frac{\partial u}{\partial t}+u\cdot \nabla u\right)=-\nabla p+\nabla \cdot \tau ,\\ \nabla \cdot u=0,\\ \frac{\partial C}{\partial t}+\left(u\cdot \nabla \right)C=\text{D}\nabla^{2}C, \end{array}$$

where *ρ* is the density of this flow (*ρ* = 1050 kg/m^3^) and **u** and *p* stand for the fluid velocity vector and the pressure. *C* and *D* (*D* = 10^+5^ *μ*m^2^/s) stand for the concentration and diffusion coefficient of sirolimus (a kind of drug released from stent struts) in blood flow [28]. *τ* is the tension tensor which is described as

(2) $$\begin{array}{c} \tau =2\eta \left(\dot{\gamma }\right)T, \end{array}$$

where $\dot{\gamma }$ and **T** stand for the shear rate and the deformation tensor rate, and the viscosity of blood is *η*. The Carreau model is used to calculate the viscosity of blood flow.

(3) $$\begin{array}{c} \eta \left(\dot{\gamma }\right)=\eta_{\infty }+\left(\eta_{0}-\eta_{\infty }\right){\left[1+{\left(\lambda \dot{\gamma }\right)}^{2}\right]}^{\left(n-1\right)/2}, \end{array}$$

where *λ* = 3.313 s, *n* = 0.3568 [29], *η*_∞_ = 3.45 × 10^−3^ kg/ms, and *η*_0_ = 5.6 × 10^−2^ kg/ms.

The article "Hemodynamic Impact of Stenting on Carotid Bifurcation: A Potential Role of the Stented Segment and External Carotid Artery" was published in 2021. Journal: Comput Math Methods Med.

*Boundary conditions for blood flow*: in this work, the boundary is as follows [15, 16, 30].

*Inlet*: the pulsatile velocity and parabolic flow velocity profile as shown in Figure 1(f) was applied at the inlet.

*Outlet*: the traction-free outflow was set at both outlets.

*Walls*: the arterial wall was treated as nonslip rigid.

*Boundary conditions for drug transport*: the simulation of drug transport was only carried out in the flowing blood.

The drug concentration value was 0 at inlet, and the mass flux of drug at the outlet and arterial wall was at 0. The drug release from stent strut was assumed in a uniform release rate (*Q* = *D*(*∂c*_stent_/*∂n*) = 1.05 × 10^−10^kg/m^2^ · s) [31].

### 2.3. Computation Procedure

The numerical simulations were conducted with the commercially available CFX (ANSYS, Inc., Canonsburg, PA, USA). Velocity-pressure coupling method was used for pressure, and the momentum equations were discretized by a pressure-based solver. Computational meshes of models in this study were obtained by ANSYS ICEM CFD (ANSYS Inc., Canonsburg, PA). Three models after stenting were meshed with tetrahedral and hexahedral elements, and near wall was with high-quality hexahedral cells. The results in this work were mesh-independent with different mesh densities. The criteria of mesh independence were set as the difference between the meshes used for computations and denser meshes which was less than 3%. To ensure the time-independent results, the 5th cardiac cycle results were presented in this article. Convergence criterion was 10^−6^ for velocity residuals and 10^−5^ for continuity.

### 2.4. Statistical Analysis

To quantitatively present the spatial distribution of WSS, the time-averaged WSS (TAWSS) during a pulsatile cycle was calculated for the data analysis, and it was defined as [32]

(4) $$\begin{array}{c} \text{TAWSS}=\frac{1}{T}\int_{0}^{T}WSS\left(s,t\right)dt, \end{array}$$

where *t* is the time, *T* stands for the time duration of a pulsatile cycle, *s* is the position on the arterial wall, and **WSS** stands for the wall shear stress vector at *t*.

The article "Hemodynamic Impact of Stenting on Carotid Bifurcation: A Potential Role of the Stented Segment and External Carotid Artery" was published in 2021. Journal: Comput Math Methods Med.

OSI is a value to evaluate the variation of WSS direction during a cardiac cycle. OSI values range from 0 to 0.5, with a high value indicating the chaos flow, and they were described as [33, 34]

(5) $$\begin{array}{c} \text{OSI}=\frac{1}{2}\left[1-\left(\frac{\left|\int_{0}^{T}WSS\left(s,t\right)\cdot dt\right|}{\int_{0}^{T}\left|WSS\left(s,t\right)\right|dt}\right)\right]. \end{array}$$

RRT is a useful parameter to measure the resident time of blood flow, indicating the regions with oscillating and low WSS. It was calculated by [33, 34]

(6) $$\begin{array}{c} \text{RRT}=\frac{1}{\left(1-2\cdot \text{OSI}\right)\cdot \text{TAWSS}}. \end{array}$$

According to the results from carotid artery study, regions exposed to “abnormal” values of TAWSS (<0.26), OSI (>0.31), and RRT (>8.95) are especially susceptible to lesion formation [34, 35]. Hence, the present study adopted these thresholds for a quantitative description of disturbed flow.

The flow ratio is defined as the peak flow of ECA to ICA during the cardiac cycle, and it was quantified as

(7) $$\begin{array}{c} \text{Flow ratio}=\frac{Q_{\max,\text{ECA}}}{Q_{\max,\text{ICA}}}, \end{array}$$

where *Q*_max,ECA_ is the peak flow of ECA and *Q*_max,ICA_ is the peak flow of ICA.

## 3. Results

### 3.1. Flow Patterns

Flow patterns in the carotid were visualized by instantaneous streamlines and contours of velocity, which were colored by the blood flow velocity magnitude (Figure 2(a)). The blood flow in the model with stenosis was characterized by significantly higher speed compared to other models, especially in the region near stenosis, ICA and ECA downstream. The narrow section had the highest velocity compared to other regions, and the blood flow kept the skewed path trajectory after the stenosis. Generally, the stented models were with evident low flow velocity in ECA and ICA. As the blood moved to the ICA, the flow was still skewed toward the outer anterior wall (Figures 2(a) and 1(e)), forming an axial velocity with crescent-shaped distribution (Figure 2, slices 1 and 2). The blood flow velocity in ICA was lower at the inner posterior wall than other regions, while the blood flow in ECA became less and in lower velocity, emerging evidently disturbed flow at the proximal ECA, and these were more obvious for the model with a medium or long stent.  Figure 2(b) shows the area of retrograde flow generated by stenting at slice 4 located at the proximal ECA. These regions were significant after the medium or long stenting. In addition, disturbed flow was observed at the distal CCA after stenting relative to the model with stenosis.

The article "Hemodynamic Impact of Stenting on Carotid Bifurcation: A Potential Role of the Stented Segment and External Carotid Artery" was published in 2021. Journal: Comput Math Methods Med.

### 3.2. Flow Distribution

To facilitate analysis of blood flow distribution after carotid stenting, the flow ratio of peak blood flow for ECA to ICA was computed. As shown in Table 1, blood flow to ECA decreased sharply after intervention, particularly as stent length increased. When a long stent is implanted, the carotid bifurcation has a flow ratio of 0.1415, which is slightly lower flow ratio as a consequence of media or a short stenting.

### 3.3. WSS Distribution

The impact of carotid stenting on TAWSS distribution was assessed. As displayed in Figure 3, TAWSS magnitude decreased remarkably at the stenting segment, particularly for the regions near struts. Moreover, the inner posterior wall of stented ICA endured abnormally low TAWSS, and the lowest value was located at the proximal stent end, while TAWSS level was considerably elevated at the downstream of stented segment. The proximal ECA and distal CCA also experienced severely reduced TAWSS, and the lowest value for each of the models was located at the outer wall of the bifurcation.

To facilitate the observation of TAWSS changes after carotid stenting, the histogram presented the area of low TAWSS level (<0.26) in Figure 4(a). As a stent was implanted, more areas with low TAWSS emerged in ICA, particularly as the stent length increased. After a long stent is implanted, the low TAWSS area was 1.45 times larger than the short one. In particular, the low TAWSS area was markedly larger in ECA compared to in stented ICA, which was over 1.65 times larger than in ICA, and this range was slightly elevated as stent length increased.

### 3.4. OSI Distribution

Figure 4(b) displays a comparison in terms of OSI for the three models after stenting. The proximal ECA could be clearly observed at relatively high OSI values. In more detail, the maximum values of OSI were located on the outer posterior wall of ECA, and this value was 0.491, 0.490, and 0.481, respectively. In addition, the inner posterior wall of stented ICA was also in high-level OSI values, particularly at the proximal stent end.

To assess the effect of stenting on the carotid bifurcation, we analyzed the area of high OSI (Figure 4(c)) statistically. The area of high OSI on the wall increased as the length of stent at ICA increased but decreased at ECA. Moreover, these areas on the ECA surface are over 11 times larger than on ICA.

### 3.5. RRT Distribution

As for RRT in Figure 5(a), it was greatly enhanced after stenting and more evident near the stent struts and bifurcation. The inner posterior wall of ICA with a stent was also in a relatively high RRT value, particularly at the proximal stent end. The maximum values of RRT in the models were located at the proximal end of ECA, and the values were 134.01, 117.806, and 67.06.

The article "Hemodynamic Impact of Stenting on Carotid Bifurcation: A Potential Role of the Stented Segment and External Carotid Artery" was published in 2021. Journal: Comput Math Methods Med.

The area of high RRT displayed in Figure 5(b) suggested that the implanted stent enhanced this value in stented ICA and ECA. Although there was little impact on the host artery, the implanted stents would induce higher RRT regions on the luminal surface of ECA than ICA. The statistical results of high RRT area on ECA wall showed that it was over 2.31 times larger than ICA.

## 4. Discussion

Emerging as a therapeutic alternative for severe stenosis, carotid stenting is still controversial due to the high rate of adverse events during follow-up. It has been evidenced that in-stent restenosis and thrombosis are the main drawbacks of this treatment [1, 4–6]. Moreover, clinical reports indicated that, in the case of carotid artery bifurcation, the implanted stent was attributed to significant stenosis that occurred in ECA after stenting [1–3, 7]. Although previous investigations provided extensive insight into the adverse events in the stented segment, they failed to quantitatively analyze the impact of stenting on the blood flow in the carotid bifurcation. This work was conducted to study the local hemodynamic characteristics of carotid stenting, exploring the potential role for adverse events after intervention.

This study found that stenting led to abnormal blood flow in the stented ICA, and the regions near stent struts were characterized by observably decreased WSS but increased OSI and RRT, especially in the inner posterior artery wall and the proximal end of the stent. These adverse mechanical parameters might explain the underlying mechanisms for clinical events, and these regions might be the primary sites to develop in stent restenosis and stent thrombosis in clinic [1, 4–6]. These numerical results presented here agreed with the early numerical conclusions [26, 30].

Moreover, our simulation results showed that the adverse mechanical conditions in the host artery after stenting may be induced by the skewed flow toward the outer anterior wall at bifurcation, and the presence of stent struts will further worsen the local blood flow. In other words, the bifurcation geometry after intervention should be given full consideration, which would probably be a key factor for the alternation of local blood flow besides the design and deployment of stents. In addition, stenting might be an alternative way to adjust the configuration and geometry of the bifurcation for improved local flow patterns.

Our numerical results also demonstrated that the implanted stents significantly reduced blood perfusion to ECA with quick restoration of ICA, and there was increased disturbed flow (retrograde flow, low WSS, high OSI, and RRT) in ECA after stenting. Moreover, the area of disturbed flow in ECA was evidently larger than that in ICA after stenting, inducing more harmful flow to ECA than stented ICA. This might severely damage ECA and significantly increase ECA occlusion after carotid stenting in clinical data [1–3, 7]. Therefore, ECA patency after carotid stenting, like recurrent stenosis and thrombosis in vessels with stents, was an important factor affecting the postoperative outcomes after intervention. These may also indicate the importance of bifurcation angles and geometry after intervention on ECA patency.

The article "Hemodynamic Impact of Stenting on Carotid Bifurcation: A Potential Role of the Stented Segment and External Carotid Artery" was published in 2021. Journal: Comput Math Methods Med.

This study also confirmed a linear relationship between abnormal flow and stent length, and long stenting would result in a larger area of low WSS, high OSI, and RRT than a shorter one. This was in agreement with clinical conclusions, which showed that the risk of in-stent recurrent stenosis and thrombosis increased with a longer stent [22, 36]. This study also indicated that the medium and long stent obviously worsen the local hemodynamic environment in ECA, implying that the long stenting induces risk for ECA intervention in clinic.

The local disturbed blood flow after stenting is a critical factor for drug transport. Our numerical results also revealed that the drug distribution in the branching model after intervention was more nonuniform (Figure 6) than that in the straight one, and the inner posterior wall near the distal part of the drug stent was in an indeed high level of drug concentration [37, 38]. This local high level of drug would seriously damage the endothelium and induce adverse events in the clinic, and the optimized performance of the stent should be designed individually for the complex artery, like branching stenting.

The sensitivity analysis due to variability of geometry and blood flow is crucial and lacking for the numerical results. Since the geometry after stenting varied with the lesions, more patients' images with different lesions should be obtained from clinical data, and postdeployment images should be performed to support our conclusions in the future. The present study only considered the stent completely implanted inside the ICA, but the stenting that covered the distal CCA to ICA is often performed for bifurcation. In that case, the stent strut would block blood flow to the ECA ostium resulting in drop in blood perfusion to the ECA; it is likely to further contribute to the branch occlusion. And also, to study the effect of stenting on the region with the stent and regions without, we ignored the stent malapposition and other problems after stent deployments, which lead to considerable disruption of flow at the region with stent [39, 40]. The present study obtained patients' images from some point of the cardiac cycle and assumed rigid wall without performing fluid-structure interaction (FSI) simulations; this might have an influence on the found results. Moreover, carotid hemodynamics is very sensitive to the boundary conditions. Results showed that different outflow conditions led to different computed intravascular pressures, while the WSS remained relatively unaffected [30, 41]. The flow split is significant to the numerical results and depends on the distal resistances, especially the minimum size of branch. In the present study, the minimum size of branch has a little difference between the models after stenting. Hence, the flow split would have limited influence on the hemodynamics in the stented carotid. Despite these limitations, the numerical results presented here agreed with the clinical data [2, 7].

The article "Hemodynamic Impact of Stenting on Carotid Bifurcation: A Potential Role of the Stented Segment and External Carotid Artery" was published in 2021. Journal: Comput Math Methods Med.

## 5. Conclusions

Stenting is an effective and widely used treatment for atherosclerotic lesions, in particular for carotid bifurcation lesions. It is now widely accepted that unfavorable blood flow has a relationship with these adverse events. The aim of the present study was to study the alterative of the hemodynamic conditions after stenting at carotid bifurcation. The numerical results showed that the implanted stent may induce an adverse hemodynamic environment both at the stented segment and the other branches without stenting, and the unfavorable alteration at ECA after stenting is much more obvious than that at the stented ICA. These indicated the occurrence and evolution of in-stent events and high risk of branch occlusion after stenting in clinic. Therefore, to achieve enhanced surgical outcome, the present results suggest that hemodynamic conditions of the vessel with stenting and the branch without after stenting are the considerable factors to achieve enhanced postoperative outcomes.

## Figures and Tables

**Figure 1:** (a) Geometry of the carotid bifurcation model with a stenosis in ICA. (b–d) Carotid models with short (13.2 mm), medium (17.7 mm), and long stent (22 mm), respectively. The locations of slices 1-6 are indicated in (c) and (d), taken as examples. (e) View of the flow presentation. (f) Inlet fluid velocity waveform [16] applied in this numerical simulation.

**Figure 2:** (a) Velocity streamlines and six representative contours of velocity in the carotid at 0.35 s. (b) Area of retrograde flow at slice 4.

**Figure 3:** Distribution of TAWSS on the carotid surface after intervention.

The article "Hemodynamic Impact of Stenting on Carotid Bifurcation: A Potential Role of the Stented Segment and External Carotid Artery" was published in 2021. Journal: Comput Math Methods Med.

**Figure 4:** (a) Area of TASS < 0.26. (b) Distribution of OSI on carotid bifurcation with a stent. (c) The surface area of OSI > 0.31 in ICA and ECA.

**Figure 5:** (a) Distribution of RRT on the carotid surface with a stent. (b) Area of RRT > 8.95 in ICA and ECA.

**Figure 6:** Distribution of drug concentration on the branching model after stenting.

**Table 1:** Effect of stenting on the peak flow rate of ECA to ICA.

	Model 1	Model 2	Model 3	Model 4
Flow ratio	0.6689	0.1425	0.1419	0.1415

## Data Availability

All data generated or analyzed during the present work are available from the corresponding author.

## Abbreviations

CCA: Common carotid artery
ICA: Internal carotid artery
ECA: External carotid artery
WSS: Wall shear stress
TAWSS: Time-averaged wall shear stress
OSI: Oscillating shear index
RRT: Relative residence time.
